The article "The Development and Usability Assessment of an mHealth Application to Encourage Self-Care in Pregnant Women against COVID-19" was published in 2021. Journal: J Healthc Eng.

# The Development and Usability Assessment of an mHealth Application to Encourage Self-Care in Pregnant Women against COVID-19

**DOI:** 10.1155/2021/9968451

**Published:** 2021-07-20

**Authors:** Khadijeh Moulaei, Abbas Sheikhtaheri, Zahra Ghafaripour, Kambiz Bahaadinbeigy

**Affiliations:** ^1^Student Research Committee, Kerman University of Medical Sciences, Kerman, Iran; ^2^Health Management and Economics Research Center, Health Management Research Institute, Iran University of Medical Sciences, Tehran, Iran; ^3^School of Health Management and Information Sciences, Iran University of Medical Sciences, Tehran, Iran; ^4^Medical Informatics Research Center, Institute for Futures Studies in Health, Kerman University of Medical Sciences, Kerman, Iran

## Abstract

The coronavirus disease 2019 (COVID-19) pandemic has caused serious concerns in pregnant women. Self-care mHealth applications can provide helpful guidelines for COVID-19 prevention or management in case of infection. This study aimed to develop and then assess a self-care smartphone-based application to provide self-care for pregnant women against COVID-19. The present study was conducted in two phases. First, a needs assessment was performed based on the opinions of 30 obstetricians and pregnant women. Then, relying on the results, a smartphone-based application was prototyped and assessed in terms of its usability and user satisfaction. To assess the application, 36 pregnant women (11 infected with COVID-19) were asked to use the application for a week. The QUIS questionnaire 5.5 was used for assessment, and the results were analyzed via descriptive statistics in SPSS 23. According to the obstetricians and pregnant women, of the 41 information requirements, 35 data elements were noted to be essential in the needs assessment. Features of the application were placed in four categories of User's Profile, Lifestyle, Disease Management and Control, and Application Functions (e.g., introducing high-risk places in terms of COVID-19 prevalence in each city, introducing specialized COVID-19 medical centers to pregnant women to receive services, medication management, stress management and control, nutrition and diet management, sleep management, contacting physicians, doctor's appointment reminder, searching the available educational materials, and making application adjustments such as text font, size, and color). With an average score of 7.94 (out of 9), pregnant women rated the application at a good level. The application can be used to reduce anxiety and stress about COVID-19 in mothers, provide access to reliable information to answer possible questions, identify high-risk locations, and provide pregnant women with instant access to healthcare facilities and information related to COVID-19 self-care processes.

## 1. Introduction

The rapid spread of COVID-19 has raised serious concerns in pregnant women [1]. Some of their major concerns are preventing and managing the disease and the potential risk of its transmission [2]. Pregnant women have a reduced tolerance to hypoxia due to their weakened immune system and physiological changes, especially in their respiratory system (e.g., lowered position of their diaphragm, increased oxygen consumption, and developed mucosal edema in their respiratory system). Therefore, when infectious diseases become epidemic, pregnant women and their fetuses become more vulnerable and highly at risk [3]. COVID-19 increases labor complications such as preterm labor, miscarriage, and fetal distress. Managing the pregnancies complicated by COVID-19 infection is challenging for physicians because there is still no consensus on issues such as optimal treatment, indications for hospitalization, choice of imaging modality, and time and route of delivery [4]. Therefore, personal protection against the coronavirus is of greatest concern to pregnant women who need special attention in terms of disease prevention, diagnosis, and management [5].

Preventing and managing the disease by use of self-care guidelines can be a promising solution to prevent or overcome respiratory diseases, especially COVID-19 [6]. Pregnancy self-care is defined as the observance of care programs and principles to ensure mothers' and fetuses' health during pregnancy, at childbirth, and in the postpartum period [7]. Self-care guidelines can be used as practical ways to reduce the possibility of infection by the coronavirus and decrease the stress caused by it [8], improve pregnant women's quality of life [9], reduce the cost of pregnancy-related healthcare, and lower the number of mortalities [10]. By following self-care guidelines, pregnant women can also avoid stress which, itself, can eliminate the possibility of weight loss in their newborns—the most significant cause of improper growth and development of infants and their mortalities [11]. McIntyre [12] believed that self-care activities during pregnancy can ensure mothers' and fetuses' health during pregnancy, childbirth, and the postpartum period. Moradi et al. [13] also investigated self-care strategies for women with gestational diabetes mellitus (GDM) during the COVID-19 pandemic and showed that following self-care programs can improve both mothers' and fetuses' health, especially among women with GDM.

In recent years, mobile technologies have been widely used to receive self-care and pregnancy care-related services. In addition to providing quick and easy access to health information, mobile applications have improved communications with healthcare systems [14]. Pregnant women have increasingly relied on social media and mobile-based health applications during their pregnancy and the postpartum period for both self-care and infant care processes and to access informative resources or receive health services. Applications can help these people to manage their health, promote a healthy lifestyle, and access reliable information at any time and place [15]. For example, low-income pregnant women were able to access personalized content (multimedia educational resources, referrals, health goals, etc.) through prenatal care coordinators (PNCCs) [16]. Tripp et al. [17] investigated pregnancy-related applications and their impact on prenatal care; they showed that pregnancy-related applications can greatly help mothers in self-care while also improving mothers' and fetuses' health. Studies have also emphasized the significance of self-care during pregnancy [18, 19] and/or during the outbreak of the COVID-19 pandemic [5, 13].

The benefits of pregnancy self-care [12], the nature of pregnancy-related applications [17], the effects of education on improving pregnancy self-care processes [20], and the evaluation of self-care strategies for women with GDM during COVID-19 [11] have all been examined in studies on pregnancy during the COVID-19 pandemic; still, it seems that no study has been conducted to develop a COVID-19 self-care application for pregnant women. Therefore, this study aimed to develop and evaluate a smartphone-based application for pregnancy self-care to help mothers protect themselves and their fetuses against COVID-19.

## 2. Materials and Methods

This descriptive-applied study was conducted in two phases. The first phase consisted of identifying and confirming self-help educational information requirements and the features required for designing the application. Based on the results of the first phase, an application was prototyped to provide self-care information to pregnant women during the COVID-19 pandemic. These phases will be elaborated as follows.

### 2.1. First Phase: Identifying and Confirming Self-Care Educational-Information Requirements and the Features Required for the Application

In this phase, the essential requirements were investigated and the required features for designing the application to facilitate self-care in pregnant women against COVID-19 were determined.

The sample consisted of pregnant women, obstetricians, and gynecologists. No sampling was performed for pregnant women. All 20 pregnant women referred to the obstetrics and gynecology ward of the 22 Bahman Health Center affiliated to Kerman University of Medical Sciences (Iran) were invited to participate, 15 of whom accepted the invitation. Moreover, all of the 15 obstetricians working at hospitals affiliated with Kerman University of Medical Sciences were invited to participate. As these physicians had experience treating pregnant women infected with coronavirus, and as they cooperated constructively with the study, the needs assessment was performed based on their opinions at this stage. The opinions of obstetricians and pregnant women were obtained using a researcher-made questionnaire, which is described hereinafter.

A five-point Likert questionnaire was designed after reviewing the relevant studies conducted on self-care against COVID-19 or its management [3, 13, 21–25] and investigating the websites of the WHO, the International OCD Foundation, and the Centres for Disease Control and Prevention (CDC) [26–28]. The questionnaire was designed to determine the required information and features for developing the application and helped collect the opinions of obstetricians and pregnant women about the significance of these needs. The questionnaire consisted of three parts: questions about the individual's demographics; questions about necessary educational informative requirements in User's Profile (8 questions), Lifestyle (6 questions), and Disease Management and Control (16 questions); and questions about their expectations about the application functionalities (11 questions). An open-ended question was also considered for each section of the questionnaire. Note that the obstetricians and pregnant women were given similar questionnaires.

Content validity ratio (CVR) was used to determine the content validity of the questionnaire. To calculate CVR, the questionnaire was given to three obstetricians and three medical informatics experts. These people had the experience of collaborating on designing self-care applications. To determine the CVR, the panel of experts was asked to answer each question based on a three-point scale (necessary, useful but not necessary, and not necessary) [29, 30]. Then, the CVR was calculated using the following formula:

(1) $$\begin{array}{c} \text{CVR}=\frac{n_{e-N/2}}{N/2}, \end{array}$$

where *n* is the number of experts who selected the “necessary” option and *N* is the total number of experts.

According to Lawshe's decision table for CVR, if the number of expert panel members is six, the minimum acceptable value for each item will be 0.99 [30]. In this study, the minimum acceptable value of CVR for each question (according to expert opinion) was 1.00. Furthermore, the total CVR ratio was calculated at 1.00. The reliability of the questionnaire was confirmed via Cronbach's alpha of 0.889 for 15 obstetricians and 0.853 for 15 pregnant women.

From July 14th to August 23rd, the questionnaire was distributed and collected among obstetricians and pregnant women. To analyze the data about educational information requirements, a scale was designed from 1 to 5 (very little, little, average, much, and very much). In addition, descriptive statistics were used to analyze the data, for which the frequency and mean were calculated. Data analysis was performed in SPSS 23. In designing the application, only those educational-information requirements and expected functions were considered which had achieved an average of 75% score (out of the total possible score) by the obstetricians and pregnant women.

### 2.2. Second Phase: Developing and Assessing the Application Prototype

First, the smartphone-based application prototype was developed based on the approved educational information requirements and the features. The application was developed via Java programming language within the Android Studio Java programming environment.

Additionally, in this phase, the problems related to application usability were identified. A virtual flyer was designed to invite the participants. This invitation was sent to a social network group that had 200 pregnant women among its members. Alongside inviting pregnant women to participate in the evaluation process of the application, the purpose and benefits of conducting the research were also explained. As a result, 41 women volunteered to participate in the study; finally, 36 women who met the inclusion criteria were selected to participate. Studies have shown that it is possible to assess the usability of an application by collecting and reviewing the feedback of 30 to 50 people, as this will reveal about 99% of the possible existing problems [31, 32]. Therefore, according to the mentioned studies, the sample size (36 pregnant women) seemed sufficient.

Inclusion criteria are as follows:

- Being pregnant
- Pregnancy >8 weeks
- Gestational age 20–50
- Absence of any underlying disease or severe pregnancy complications and risk factors for childbirth identified based on the family's health records or the pregnant woman's claims
- Pregnant women who did not need special care or partial/absolute rest
- Being literate
- Using smartphones daily
- Consenting to participate

Exclusion criteria are as follows:

- Pregnant women's illness and poor physical/mental condition
- Pregnant women's reluctance to continue participation

In the next step, the application was sent to the participants along with its installation guide on their mobile phones. After confirming that the application had been successfully installed on the participants' mobile devices, they were asked to use the application. To ensure that the participants were using the application, a message was sent to them on a daily basis with the following content: “Please do not forget to use the application.”

After a week, the participants were asked not to use the application anymore. Then, by using the standard Questionnaire for User Interface Satisfaction (QUIS), their opinions were asked about the usability of the tool and whether they were satisfied with it [33]. Like previous studies [34], the validity of QUIS was confirmed in this study and its reliability was evaluated and confirmed by Cronbach's alpha (0.92).

The QUIS questionnaire has six parts: three questions addressing the identity of the participants, six questions about the overall reaction to the app, four questions related to the screen, six questions related to the terminology and information used in the application, six questions related to the learning, and five questions dealing with the app's capabilities. This questionnaire was designed based on a 10-point Likert scale. The mean scores of 0–3 were classified as poor, 3.1–6 as intermediate, and 6.1–9 as good.

The data were analyzed using descriptive statistics, including mean and standard deviation in SPSS 23.

## 3. Ethical Considerations

Ethics approval (IR.KMU.REC.1399.240) was obtained from the Ethics Committee of Kerman University of Medical Sciences. The obstetricians' and pregnant women's participation was voluntary, and the individuals were free to withdraw from the study at any time. Informed consent for participation was obtained from the participants. For all pregnant women, the use of the application was free of charge during the assessment process. Data collected from pregnant women (whether infected by the coronavirus or not) were used without identifying their personal information.

## 4. Results

### 4.1. Self-Care Educational-Information Requirements and the Features Required for the Application

Table 1 shows the demographic details about the participants. Most obstetricians were 30–40 years of age and had 1–5 years of work experience. Among the pregnant women, 80% had had 1-2 pregnancies, and two women had COVID-19 (13.33%) at the time of the study.

The findings related to the educational information requirements were divided into four categories: “User's Profile, Lifestyle,” “Disease Management and Control,” and “Application Functions.” The participants' opinions about the necessity of applying certain features are presented in Table 2. In recording the participants' demographic information in the User's Profile, the individuals' national ID number, age, weight, and height were not included as the participants had rated the necessity of this information less than 75%. In Lifestyle, information related to exercising was excluded. As for the other cases, the participants believed that recording information about the User's Profile, Lifestyle, Disease Management and Control, and also Application Functions was necessary.

### 4.2. Designing and Assessing the Mobile-Based Application Prototype

The application was designed based on the results obtained in the first stage (Figure 1). In the “User's Profile,” pregnant women should enter and save their demographic information. In the user's “Lifestyle” section, some advice and educational self-care information is provided to help pregnant women to avoid COVID-19. In the “Disease Management and Control” section, COVID-19 is introduced and explained to pregnant women and medical guidelines are provided on how to manage and control the disease based on valid academic resources and specialists' recommendations.

In the COVID-19 “Symptoms” section, just by entering certain information about symptoms such as dry cough, fever, chills, sore throat, shortness of breath, body temperature, and possible underlying diseases, pregnant women were informed whether they were infected with the coronavirus or not (Figure 2). In the “Introducing high-risk areas in the city” section, where high-risk places (in terms of a high prevalence of COVID-19) were introduced to the pregnant users, the areas where the risk is considerably alarming were stated so that the users would avoid going to those places. Also, in the section where specialized healthcare centers were introduced, the users were provided with information about the locations of all these centers throughout Iran in case they needed to receive certain medical services (Figure 3).

In the “Medications Management” section, it was possible to record the names of the medications, their doses, and their timely intake schedule, and it was also possible to view the list of reminders and previous medications. In “Stress Management and Control,” some videos and educational materials were provided to help pregnant mothers reduce and manage their stress. In “Nutrition and Diet Management,” pregnant mothers were allowed to plan a proper diet to help them strengthen their immune system and increase their body resistance against COVID-19. In “Sleep Management,” the user could control and manage her sleeping time and duration. In “Contacting Physicians,” a list of names, contact information, and office or treatment center addresses were provided in case the user required further consultation on COVID-19 and its effects on their pregnancy. In “Doctor's Appointments,” users were able to handle all the items required to arrange a doctor's appointment.

In “Search,” the users could search for educational materials to gain more information about pregnancy, mothers, fetuses, and COVID-19. In “Settings,” the users could manage the font type, size, and color of the presented materials. Further details on each section along with related illustrations are provided in Appendix.

The usability and user satisfaction with the self-care application were evaluated. The demographic information of the pregnant women participating in this stage is presented in Table 3.

The results of the usability evaluation using QUIS are presented in Tables 4 and 5.

Table 4 demonstrates pregnant women's opinions in assessing the self-care application, along with the mean and standard deviation obtained from analyzing the data. In all the assessed aspects, an average of >6 was achieved; thus, it seems that the users generally believed that the application was good. Information about each of these aspects is provided in Table 5.

## 5. Discussion

We developed a smartphone-based application to facilitate pregnant women's self-care against COVID-19 and evaluate its usability. Based on the opinions of the specialists and pregnant women, most of the data elements, educational information needs, and functions were approved. Moreover, the User's Profile and Lifestyle information (excluding the data about patients' age, weight, height, education level, exercise, and national ID number) was approved. The five dimensions of usability scored an average of >6, indicating that users rated the application at a good level. Table 5 compares the results of the present study to related studies.

In this study, similar to other studies, educational needs could be provided to pregnant women through different methods such as texts, educational videos, audios, and images regarding all three dimensions of “Lifestyle,” “Disease Management and Control,” and “Application Functions.” Nussbaum et al. [35] stated that mHealth applications have numerous functions and offer various features to help with disease management, such as home-based exercise programs, symptom trackers, medication diaries, educational information, and movement analysis. Dasuki and Zamani [36] also stated that mobile phones can be used to improve mothers' and pregnant women's maternal health literacy instead of merely being used for accessing maternal healthcare. Oyeyemi and Wynn [37] believe that mobile phones provide a platform for pregnant women to stay connected to one another and freely share their health-related issues with midwives; consequently, this will help promote their self-confidence and self-esteem and raise the possibility of applying maternal practices that have been confirmed and recommended in other studies. In most of the studies listed in Table 6, providing information related to the pregnancy period for pregnant women has been greatly taken into consideration as the most important educational requirement to help increase pregnant women's health knowledge [16, 38–42].

In the present study, as in other studies, pregnant women could set reminders to keep track of their doctor's appointments, medication schedule, and their fruit and vegetable intake. According to Table 6, reminders have been considered as one of the most important features in these studies [16, 38, 42]. In the literature, different purposes such as follow-ups [16], daily loggings, information about pregnancy weeks [38], and sending appointments [42] have been mentioned for reminders. Various studies have shown that the use of reminders can have a positive impact on patient appointment attendances [43], adherence to using the drugs [44], antiretroviral therapy [45], patient self-management [46], and improving health outcomes and patient care processes [47].

Three randomized clinical trials (RCTs) reviewed antenatal care (ANC) services and concluded that the use of appointment reminders and prenatal training for pregnant women can play a significant role in encouraging mothers to visit their physician or care-provider regularly, improving mothers' knowledge and understanding, and enhancing their health status [48–50]. Entsieh et al. [51] investigated the significance of sending reminders to pregnant women to remind them of planned antenatal care visits and reported that reminders could increase planned antenatal care visits.

The application presented in the present study has other functions such as introducing high-risk places (i.e., with a high prevalence of COVID-19) in each city, introducing specialized COVID-19 medical centers to pregnant women to receive required services, COVID-19 symptoms and diagnosis, drug management, stress reduction and control, nutrition and diet management, sleep management, contacting physicians, searching related educational materials, making application adjustments (e.g., font type, size, and color), and providing specialized information about women's self-care practices, provided in the two categories of Lifestyle and Disease Management and Control.

Because the present study focused on pregnant women's self-care against COVID-19 during their pregnancy, the functions such as high-risk locations in each city, introducing COVID-19 specialized medical centers, and COVID-19 diagnosis are completely different from those listed in Table 3. Furthermore, all the educational information contents of this application have been presented with a focus on encouraging proper self-care in pregnant women against COVID-19 during their pregnancy.

Herein, after identifying the educational needs and required functions of a reliable self-care application for pregnant women, the application was designed and its use was assessed. Usability assessment was performed with the cooperation of 36 pregnant women (11 pregnant women who had had COVID-19 and 25 who had not been infected). The assessment results showed that the users were well-satisfied with the application.

As observed in Table 5, previous studies have applied different methods to assess the usability of applications. Keedle [39] evaluated the system to assess users' ability in completing the assigned tasks. In this study, a web-based survey was performed to assess the usability of the designed application.

Hussain et al. [40] assessed five usability dimensions, namely, effectiveness, efficiency, learning ability, memorability, and satisfaction, based on Jakob Nielsen's usability principles. Moreover, van Beukering et al. [41] applied the think-aloud protocol to identify the application's flaws which were then ranked based on Nielsen's severity scale. The findings of all these studies have indicated that different assessment processes can identify and resolve relevant problems. The most common issues identified in these studies were utility (e.g., failing to provide a “forgot password” button), terms and information used in the application (e.g., when displays were required to appear more than once, the application failed to show the message at the proper time) [39], terminology interpretation problems, unclear and incomprehensible buttons, finding and understanding work advice [41], and memorability (e.g., understanding the displayed icons, locating the provided information, refinding it, and navigating through the mobile app) [40]. In the present study, most of the identified problems were mainly related to learning capabilities and the terminology and information used in the application.

The limited number of participants in the needs assessment and evaluation and the short duration for evaluation are the limitations of this study. This was, however, due to the conditions of the COVID-19 pandemic and the urgency to design and evaluate a helpful application. Other studies have also encountered comparable challenges [16, 38]. Therefore, it is recommended that the same study be conducted on more specialists and pregnant women, over a longer period, to further reveal the merits and possible flaws of the application, as well as new users' requirements and expectations. Moreover, the designed application's effectiveness in improving pregnant women's self-care behaviors and health status has not been evaluated, which is another limitation that will be investigated in future studies.

The application presented here was designed and evaluated based on scientific documents and the opinions of obstetricians and pregnant women. Our application offers different services (e.g., introducing high-risk places in terms of COVID-19 prevalence in each city, introducing specialized COVID-19 medical centers to pregnant women to receive services, medication management, stress management and control, nutrition and diet management, sleep management, contacting physicians, doctor's appointment reminder, searching the available related educational needs, and making application adjustments such as font type, size, and color) for women during prepregnancy, pregnancy, and postpregnancy (breastfeeding) periods. In other words, this application helps pregnant women in two ways; first, it is a tool for tracking pregnancy and its changes, and second, it increases the awareness of pregnant women about their health and issues related to pregnancy and beyond during the COVID-19 outbreak. Therefore, it can be widely used by pregnant women to alleviate their concerns about COVID-19 and maintain maternal and fetal health.

In the future, we intend to examine the impact of this application on pregnant women through a case-control study. We also plan to add some new capabilities to the app, such as electronic pregnancy records and face-to-face communication with obstetricians. These capabilities reduce the need for pregnant women to visit medical facilities in person and thus decrease the risk of COVID-19 transmission.

## 6. Conclusion

This study developed and assessed a mobile-based self-care application for pregnant women to help protect them against COVID-19. This application can provide various services to reduce maternal anxiety and stress about COVID-19, allow quick diagnosis of COVID-19, reduce the possibility of infection, provide rapid access to reliable answers for possible questions, identify high-risk locations (in terms of COVID-19 prevalence) in every city of Iran, provide pregnant women with instant access to COVID-19 healthcare centers and information about coronavirus, and explain self-care and self-management processes. The assessment of the application's usability also showed that users evaluated the application at a good level. Therefore, this application was considered as a prototype, a model for designing other similar applications that provide self-care against the coronavirus. With daily use of this easily accessible self-care application, pregnant women are allowed to personally monitor their health and help control and prevent COVID-19.

## Figures and Tables

**Figure 1:** The main page of the self-care against COVID-19 application for pregnant women.

**Figure 2:** Diagnosing COVID-19.

**Figure 3:** All specialized COVID-19 treatment centers in Iran.

**Figure 4:** Medication reminder.

**Figure 5:** Stress management and control.

**Figure 6:** Doctor's appointment.

**Table 1:** Demographic information of the participants of the first phase.

Variable	Frequency	Percent
Obstetricians		
Age (year)		
30–40	9	60
46–51	6	40
Work experience (year)		
1–5	7	46.6
6–11	3	20
>11	5	33.3

Pregnant women		
Age (year)		
20–30	8	53.3
31–40	5	33.3
40–50	2	13.3
Education level		
High-school diploma	3	20
Bachelor's	7	46.6
Master's	5	33.3
Infected with COVID-19		
No	13	86.6
Yes	2	13.3
Number of pregnancies		
1-2	12	80
3-4	2	13.3
≥5	1	6.6

**Table 2:** Obstetricians and pregnant women's opinions about the necessity of educational information requirements and application functions.

Categories	Data elements	Obstetricians' perspective	Pregnant women's perspective
		Average answers in percent	Average answers in percent
User's Profile	Name and surname	89	84
	National code number	65	54
	Age	69/22	31
	Weight	74	44
	Height	73	21
	Education	65	54
	Residential address	87	76
	Contact number	90	89

Lifestyle	Exercise	72.4	65.2
	Sleep	89.54	78.9
	Having proper nutrition during the COVID-19 pandemic	90.8	77.21
	Smoking, drinking alcohol, and using hookah while pregnant and/or during the COVID-19 pandemic	81.6	76.65
	Managing stress in pregnant women during COVID-19 pandemic	93.4	89.9
	Motivational messages	93.4	91.2

Disease Control and Management	Introducing and explaining COVID-19 to pregnant women	86.1	79.43
	COVID-19 symptoms	83	91.22
	COVID-19 side effects	83	92.3
	The transmission of COVID-19 from the mother to the fetus	81.6	94.2
	COVID-19 in pregnancy and nursing	86.1	91.34
	Avoiding COVID-19	86.2	87.37
	Observing personal hygiene (e.g., proper handwashing training and alcohol use)	86.2	78.4
	Respiratory health	81.6	76.65
	Proper contact methods for connecting with others	80	78.68
	The dangers of using masks, alcohol, and other preventive methods for pregnant women	81.6	93.44
	Avoiding stressful relations and environments	86.8	94.3
	Maintaining proper nutrition and diet during the COVID-19 pandemic	90.8	77.21
	Maintaining mental health	93.4	89.9
	Primary measures to be taken when infected with coronavirus	88.67	98.2
	Home quarantine	85.44	77.39
	Receiving reliable information and news	79.02	76.12

Application Functions	Primary diagnosis of COVID-19 in pregnant women	86	86.8
	Introducing high-risk areas in the city (where there is high COVID-19 prevalence)	85.6	78.4
	Introducing specialized COVID-19 medical centers to pregnant women who seek care	84.67	79.21
	Managing medication intake	87.6	79.29
	Reducing and controlling stress	93.4	89.9
	Managing nutrition and diet	90.8	77.21
	Managing sleep	80	78.68
	Contacting a physician	88.45	98
	Doctor's appointment reminder	86.29	78.3
	Searching in available educational material	78.21	76.35
	Application settings (text size, font, color, etc.)	86.33	80.01

**Table 3:** Demographic information of pregnant women.

Variable	Frequency	Percent
Age		
20–30	17	47.22
31–41	14	38.88
41–50	5	13.88

Education level		
High-school diploma	5	13.88
Bachelor's	28	77.77
Master's	3	8.33

Infected with COVID-19		
No	25	69.44
Yes	11	30.55

Number of pregnancies		
0-1	22	61.11
2-3	9	25
≥4	5	13.88

Month of pregnancy		
1–3	12	33.33
4–7	19	52.77
8-9	5	13.88

**Table 4:** Assessing the self-care application's usability and user satisfaction.

Assessed aspects	Mean (±SD)
Overall reaction to the app	8.07 (±1.26)
Screen	8.13 (±1.17)
Terminology and information used in the application	7.51 (±1.20)
Leaning	7.49 (±0.78)
App capabilities	8.62 (±0.81)
Total	7.96 (±1.04)

**Table 5:** Results of assessing different aspects of the application.

Assessed aspects	Questions about each aspect	Mean (±SD)
Overall reaction to the app	General use of the application	8.31 (±1.01)
	Ease of use of the application	8.28 (±1.11)
	How the user feels about using the application	7.49 (±1.62)
	General design of the application	7.21 (±0.98)
	Consistent use of the application	8.69 (±1.43)
	The settings feature of the application	8.48 (±1.41)

Screen	Reading characters on the screen	8.01 (±1.02)
	Using clear statements to simplify tasks	8.42 (±0.98)
	Organization of information	7.69 (±1.81)
	Sequence of screens	8.40 (±0.89)

Terminology and information used in the application	Use of terms throughout the system	7.21 (±1.38)
	Task-related terminology	7.43 (±1.65)
	Position of messages on the screen	8.48 (±1.34)
	Prompts for input	7.42 (±1.18)
	App messages to complete user's tasks	7.13 (±0.78)
	Error messages	7.43 (±0.89)

Learning	Learning to operate the system	7.41 (±0.68)
	Exploring new features by trial and error	7.13 (±0.79)
	Remembering names and use of commands	7.48 (±0.61)
	Straightforward task performance	8.42 (±0.89)
	Help messages on the screen	7.02 (±0.98)
	Supplemental reference materials	7.52 (±0.77)

App capabilities	App speed	8.61 (±0.92)
	System reliability	8.70 (±0.73)
	Number of app specifications	8.59 (±0.86)
	Correcting user's mistakes when inputting data	8.42 (±0.68)
	Designed for all levels of users	8.78 (±0.79)

**Table 6:** Features mentioned in previous studies.

Ref.	Aim of the study	Information-educational needs and application functions	Type and purpose of evaluation	Number of people participating in the evaluation
Chaudhry et al. [16]	To design, develop, and evaluate an application for low-income pregnant women	Referral follow-up and tracking, data sharing among health actors, calendar and reminders for pregnant women to follow up with prenatal care coordinators (PNCCs), trackers for specific health indicators, educational library	To evaluate the usability of the application for the target population by evaluating their ability to perform the assigned tasks	9 pregnant women

Sajjad and Shahid [38]	To support pregnant women in Pakistan to track their pregnancies and control them more	(1) A personal health record system customized by the user during pregnancy and approved by a gynecologist. In this system, women can (1) record their health data (gaining weight over time, etc.), (2) a module for prayers, Quranic verses and verses for daily support, (3) logging in to the system for tracking weight and daily food intake, e.g., through fruits and vegetables per day, (4) a module related to answering local myths and common Islamic FAQs, (5) exercise program (recommended by a gynecologist based on women's condition and stage of pregnancy), (6) exercise section, (7) pressure notification system for various tasks (daily login reminders, pregnancy week information, etc.), (8) Baby tracker, and (9) quick guide (tips) to stop women from high-risk behaviors	A usability test to evaluate the usefulness and acceptance of the application	14 pregnant women

Keedle et al. [39]	The development and evaluation of a smartphone mobile software application (app) to collect qualitative data of the pregnant women	Creating an account, creating an audio or video log, uploading a log	The evaluation included installation, signing up, recording a log, uploading a log, appearance, and improvement	7 pregnant women

Hussain et al. [40]	Evaluation of the ease of use of a mobile app interface to ensure pregnant women and their spouses about the usability of the application	Weekly follow-up of pregnancy status, learn about the baby, calculate the current week of pregnancy, calculate the due date (date of pregnancy), track your weight, track your baby's beats, keep notes of pregnancy symptoms (morning sickness), change in the body, doctor's appointment	Evaluating the five dimensions of usability: Effectiveness, efficiency, learnability, member ability, and satisfaction according to the principles of usability (Jakob Nielsen)	15 pregnant women and their husbands

van Beukering et al. [41]	Usability of the mHealth pregnancy and work app and the perceived usefulness of the work advice, the main goal of the app, by potential end-users	Information and advice about work-related pregnancy risks	Usability evaluation based on the intrinsic motivation inventory (IMI) score and the system usability scale (SUS)	12 working pregnant women

## Data Availability

No data were used to support this study.

## Appendix

### Details about Different Modules of the Designed Application

In “User's Profile,” besides entering demographic data, a pregnant woman can upload her picture and edit her information whenever she desires. The “Lifestyle” section includes necessary self-care advice and training for developing healthy sleeping habits, developing proper nutrition plans during the COVID-19 pandemic, avoiding smoking, drinking alcohol, and using a hookah, managing stress in pregnant women during the pandemic, and sending motivational messages. This module has been developed for physical, mental, and spiritual self-care. In “Disease Management and Control,” different aspects of COVID-19 during pregnancy are introduced and some methods for self-care are suggested to prevent COVID-19 infection. Individuals are encouraged to follow the presented hygiene protocols.

Pregnant women can record symptoms such as dry coughs, fever, chills, sore throat, shortness of breath, body temperature, and underlying diseases in the application, and it will allow them to find out whether they are infected with the coronavirus. Based on the entered information, if the application recognizes that the user is or may be infected with the coronavirus, a message will appear on the screen stating, “Visiting a medical center is advised” (Figure 3). Informing users about high-risk locations (in terms of the prevalence of COVID-19) in each city was designed to help pregnant women avoid going to those locations. Here, the user can select a province, city, and street of residence. “Locations with a high risk of COVID-19 prevalence” are displayed in red to prevent possible traveling to those locations.

As for “Introducing Specialized COVID-19 Medical Centers” in the application, the locations of all of these medical centers in Iran are provided so that it would be more convenient for pregnant women to receive the care and services they need within their own region (Figure 3). By clicking on each city or hospital available on the map, all the necessary information is displayed.

In “Medications Management,” in addition to the functions introduced in the main text (Figure 4), pregnant women can also enter their physical health information such as their heart rate, blood pressure, and blood sugar, even when these are abnormal. They can also share this information with their physician to receive more effective treatment.

In “Stress Management and Control” for pregnant mothers, the level of stress can be determined on a scale of low, medium, and high (Figure 5). By selecting medium or high levels of stress, a number of motivational and positive messages will appear on the screen and some educational videos on reducing stress levels will be suggested. Additionally, in this section, the user can receive a report on the number of stressful days that they have experienced within different time spans and the results are also displayed on a graph.

In “Nutrition and Diet Management,” users can plan a proper weekly diet. The application also reminds them to intake fruits and vegetables, while at the same time, keep track of the food consumed in every meal and the number of calories received. The application also displays videos about nutrition and maintaining a healthy diet during pregnancy (as advised by specialists). Furthermore, by recording the user's diet and daily exercise activities or even daily steps, the application can allow the user to keep track of their weight loss or gain by observing their changes on displayable charts.

In “Sleep Management,” users can record the time at which they wake up, plan a regular sleep pattern, and receive a report on their sleeping status (how long they have slept per day, week, and/or month) within different time intervals.

In “Contacting a Physician,” a list of physicians' names, contact information, and office locations at medical centers is provided. If necessary, a pregnant woman can receive advice from these physicians either by phone or by in-person visits. The physicians listed in this application had consented to cooperate to help prevent the further spread of COVID-19 and reduce its threat to mothers and their babies.

In the “Doctor's Appointment Reminder” section, the pregnant woman is given the opportunity to record the date of the doctor's appointment, his/her name and location at a medical center, and a description stating the purpose of the appointment. Based on the arranged date, the application sends the user a reminder of her doctor's appointment which is displayed on the screen (Figure 6).
